# Image Enhancement Technology Based on Deep Trust Network Model in Clinical Treatment of Traumatology and Orthopedics

**DOI:** 10.1155/2021/1717512

**Published:** 2021-07-10

**Authors:** Qiaomu He, Shenghao Chen, Lei Li

**Affiliations:** Suizhou Hospital, Hubei University of Medicine, Department of Orthopedics, Hubei, Suizhou 441300, China

## Abstract

Fractures have brought great pain to patients, and treatment requires a lot of time and yield slow results, which seriously affect the production and life of people. Fractures are mostly treated with traditional conservative treatment methods. For orthopedic trauma, image enhancement technology has gradually played an important role in the clinical treatment of orthopedic trauma and has become a kind of suffering. It has become a new treatment method that attracts people's attention. In order to study the application of image enhancement technology based on the deep trust network model in the clinical treatment of trauma and orthopedics, this paper conducted a related survey of fracture patients in the city's first hospital, reviewed relevant literature, and interviewed professionals, and we collected relevant material, constructed case templates, and created clinical research models using comprehensive quantitative and qualitative analytical techniques. Studies have shown that the use of image enhancement techniques in the treatment of fractures has been successful, with healing efficiency approximately 20% faster than conservative treatment. In the clinical treatment of trauma and orthopedics, image enhancement technology can effectively reduce the incidence of complications in the prognosis of patients. *Symptom Drop.* This shows that the image enhancement technology of the deep trust network model can play an important role in the clinical treatment of trauma and orthopedics.

## 1. Introduction

Deep venous thrombosis (DVT) is one of the most common peripheral vascular diseases in clinical practice, referring to impaired venous return caused by abnormal deep venous blood clotting [1]. This mainly occurs in the lower extremities and is a clinical emergency. The incidence of deep vein thrombosis in patients with traumatic fractures is very high. Plastic surgeons should pay attention to this and take appropriate preventive measures. Although DVT has received high clinical attention, most patients who are bedridden due to fractures are still receiving conventional anticoagulation therapy, but based on anticoagulation therapy, many patients still have DVT. Compared with previous studies, DVT in orthopedic trauma has been reduced. However, in recent years, with the increasing importance of DVT, posthospital coagulation therapy has become increasingly standardized, but the incidence of DVT in orthopedic patients has not decreased significantly. This problem deserves our attention [2].

With the aging of the world population and changes in people's lifestyles and habits, venous thromboembolism (VTE) caused by trauma and orthopedics has become an increasingly serious global health problem. It is an academic problem internationally and has attracted social attention. VTE is a common disease with high morbidity and high mortality. In the United States, the incidence rate is higher than stroke and myocardial infarction, and the death rate is much higher than breast cancer and AIDS. It is considered the second largest unemployed population. With upper respiratory tract infection [3], the disease causes enormous financial and energy burden on society and families. Therefore, the prevention and treatment of VTE is an important topic that must be paid attention to clinically and socially [4].

For the treatment of trauma and orthopedics, experts at home and abroad also have conducted a lot of research. Argaw et al. evaluated the practice of surgical antimicrobial prevention (SAP) and surgical site infection (SSI) based on the review of the medical records of patients undergoing surgery in the orthopedic and trauma surgery of the Tikkul Ambesar Specialist Hospital (TASH). Antimicrobial prophylaxis was carried out for patients, which achieved some effect in orthopedic trauma treatment [5]. Vaishya et al. evaluated the fixation technology using preformed locking plates to understand whether it provides stable fixation and has a good functional outcome. A total of 32 patients with fractures of the lateral end of the clavicle (Neer type II) were included. After obtaining informed consent and performing preoperative examination, under general anesthesia, a 3.5 mm precontoured upper locking plate was used to extend laterally for open reduction and internal fixation. It is proved that the fracture becomes unstable due to various deformation forces acting on the fragments and the distal small fracture fragments [6]. Yoda et al. believe that fractures can be treated with high-frequency ultrasound. Based on fracture statistics entered at the University Medical Hospital, a control experiment was performed in which fracture sites were formed in fracture patients using high-frequency ultrasound, and the fracture sites were targeted and guided. It can be fastened with inner nails to reduce and heal fractures [7]. Nyland et al. believe that traditional Chinese medicine has a specific effect on fracture prognosis. The prognosis of fractured patients is treated with traditional methods of fumigation of herbal medicines. High‐frequency ultrasound was used to guide the fracture site. Experimental results show that smoking, a traditional herbal medicine, significantly improves the patient's blood flow rates, reduces serum levels, and benefits the prognosis of patients with fractures [8].

In this article, with the introduction of a deep trust network model, the therapeutic effect of image enhancement technology in clinical trauma and orthopedics is compared with other orthopedic treatment methods. The role of image enhancement technology in trauma and orthopedics is compared with the collection of relevant experimental data. The comparative results of the experimental data were analyzed in more detail and multilevel. Finally, it was concluded that based on patient and expert tests, the experimental conclusions showed that image enhancement technology has high practical value in orthopedics trauma.

## 2. Application Methods of Image Enhancement Technology in Clinical Treatment of Trauma and Orthopedics

### 2.1. Deep Trust Network Model

The deep network of trust is formed by a large number of artificial neurons. Humans use computer technology to simulate and perform the functional connection of biological neurons. It has the properties of a nonlinear (dynamic) system. The deep trust network also has the characteristics of high dimensionality (composed of many neurons, multiple input-multiple output), parallelism, distribution, self-adaptation, self-organization, and self-learning capabilities [9, 10]. A single neuron is not complicated, but a deep trust network composed of a large number of neurons can produce extremely complex and extremely rich phenomena and results [11].

Generally speaking, the traditional trust network model algorithm is as follows:

(1) $$\begin{array}{c} G\left(x,y\right)=\exp\left(-\frac{x^{2}+y^{2}}{2\sigma^{2}}\right), \end{array}$$

where *σ* is means square error. It is achieved by kernels and convolutions with different *σ* values. The resulting expression formula is as follows:

(2) $$\begin{array}{c} L\left(x,y\right)=-\frac{1}{\pi \sigma^{4}}\left(1-\frac{x^{2}+y^{2}}{2\sigma^{2}}\right)\exp\left(-\frac{x^{2}+y^{2}}{2\sigma^{2}}\right). \end{array}$$

The effect is related to the value of *σ*

(3) $$\begin{array}{c} Q=\frac{1}{2a^{2}r^{-1}}{\left(\frac{2b^{2}}{a^{2}r^{-1}}p-t\right)}^{-1}\left[a^{2}r^{-1}t^{2}+2\left(1-b^{2}\right)t\right], \end{array}$$

where *a* ∈ [−1,0] ∪ [0,1]:

(4) $$\begin{array}{c} K=\frac{a}{2br}t, \end{array}$$

(5) $$\begin{array}{c} \lambda_{x}\left(ct_{n}-t\right)>0, \end{array}$$

and so

(6) $$\begin{array}{c} Q=\frac{1}{2a^{2}r^{-1}}{\left(\frac{2b^{2}}{a^{2}r^{-1}}t-L\right)}^{-1}\left[a^{2}r^{-1}L^{2}+2\left(1-a^{2}\right)L\right]. \end{array}$$

The deep trust network is a multidimensional spatial interpolation technology, which overcomes some shortcomings of the traditional trust network model and has a wide range of uses. The deep trust network is a mathematical model that can simulate synaptic agglutination in the brain, which is very similar to the structure of the human brain, and has powerful functions to deal with nonlinear approximation problems and features [12]. The radial base neural network is a supply neural network. It has powerful editing capabilities for nonlinear problems, is not easy to optimize locally, has a simple structure, can solve complex problems, and is easy to train. Learning converges quickly. The deep trust network has strong self-learning ability, can approximate any nonlinear function, and responds well to data changes. The entire input and output process of the deep trust network is roughly as follows: first, the nonlinear mapping from the input layer to the hidden layer and then the linear mapping from the hidden layer to the output layer [13]. The structure of the deep trust network is shown in Figure 1.

The parallel processing function of deep trust network effectively guarantees its data processing efficiency. The deep trust network separated from the hierarchical structure is a forwarding network consisting of an entry level, a hidden level, and an exit level. The input level configuration consists of source nodes, the hidden level is defined by the user according to specific real conditions, and the output level is a specific response to the input level [14]. The number of neurons in the hidden layer is usually determined by the golden section optimization method. After clearing the number of neurons, you can skip the link and map the input vector directly to the hidden layer. The process is shown in Figure 2:

The deep trust network algorithm is as follows:

(7) $$\begin{array}{c} \langle u\rangle =\int_{-\infty }^{\infty }u{\left|F\alpha \left(u\right)\right|}^{2}\text{d}u=\int_{-\infty }^{\infty }f*\left(t\right)\varepsilon^{a}f\left(t\right)\text{d}t, \end{array}$$

where *ε*^*a*^ represents the fractional frequency operator, and its expression is

(8) $$\begin{array}{c} \varepsilon^{a}=\cos\;\alpha *\delta +\sin\;\alpha *\lambda . \end{array}$$

In the formula, *δ* is a time operator and *λ* is a frequency operator. Using the relationship with the instantaneous variable, the instantaneous fraction *u* of *s*(*t*) can be expressed as

(9) $$\begin{array}{c} u\left(t\right)=\kappa \left\{\frac{\gamma s\left(t\right)}{s\left(t\right)}\right\}. \end{array}$$

Substituting into the formula, we can get

(10) $$\begin{array}{c} u\left(t\right)=\kappa \left\{\frac{\lambda s\left(t\right)}{s\left(t\right)}\right\}=\kappa \left\{\frac{\cos\;\alpha *t*s\left(t\right)+\sin\;\alpha *\left(-jds\left(t\right)/\text{d}t\right)}{s\left(t\right)}\right\}. \end{array}$$

The parallel processing capability of the deep trust network can be expressed as

(11) $$\begin{array}{c} r\left(t\right)=d\left(t\right)s\left(t\right)=d\left(t\right)\text{rect}\left(\frac{t}{T}\right)e^{jwbt}. \end{array}$$

The image enhancement technology after the introduction of the deep trust network can effectively improve the application of orthopedic trauma in patients' imaging and provide assistance for treatment.

### 2.2. Traumatology and Orthopedics Characteristics

Bone damage is mainly caused by high energy damage. Such patients are seriously ill and develop rapidly. Due to the possible lesion, there were no clinical symptoms at that time. Therefore, it is more difficult to diagnose patients and it is easier to miss the diagnosis [15]. Due to the different injured parts, the severity of organ and limb injuries is inconsistent, the sequence of rescue operations is also different, and the focus of treatment is also inconsistent, so it is easy to avoid serious or minor injuries. From the survey, we can see that the main reason is injuries caused by car accidents and falls. In the case of limb impact, impact, pressure, etc., the limbs, pelvis, and spine are the main stress points, so even if they are opened, they are easy to fracture [16].

In addition to fractures, patients often suffer injuries to other parts of the body, mainly the chest, abdomen, and brain. In addition, the patient's hemodynamics at admission is very unstable [17]. Severe fractures can cause the surrounding organs and skin to rupture, thereby damaging soft tissues and major blood vessels, and making them more susceptible to traumatic hemorrhagic shock. Other parts, especially head injuries, are common injuries. Such patients are prone to acute traumatic coagulopathy (ATC) due to persistent bleeding or open injury or vascular injury. Its physiological functions can cause hypotension, acidosis, and blood clotting. The immune response is in a state of high pressure, leading to dysfunction, hypofunction, and hypothermia, as well as an abnormal immune inflammatory response after trauma. Inflammatory factors produced by macrophages, neutrophils, and other effector cells activate the innate and endogenous immune system to form a “cascade effect” [18]. And, it develops into a severe systemic inflammatory response syndrome (which can lead to SIRS) and further leads to multiple organ failure (MOF).

Traumatic stress can cause systemic inflammatory response syndrome (SIRS) and increase the body's sensitivity. Severe open wound infection and long-term use of various invasive catheters, combined with an increased incidence of internal infections, can lead to drug resistance. Anti-infective bacteria may lead to the risk of ineffective antibiotic treatment. Therefore, multiple injuries have the following clinical characteristics: (1) high infection rate; (2) significant increase in the incidence of shock; (3) severe stress response; and (4) high complications and mortality. Therefore, to consider which surgical method and how to treat multiple severe fractures, the patient's resistance to the second blow must be considered. The traditional surgical method is the early and direct repair of fractures, which requires stripping of tissue and periosteum to reduce and repair fractures. Blood loss is also obvious, and the patient's blood volume is significantly reduced [19]. This can irritate the body and cause systemic vasospasm. In addition, frequent blood transfusions and blood transfusions will lower the patient's body temperature and cause the blood coagulation mechanism to fail. Therefore, by using image enhancement technology to image the injured part of the patient, the injured state of the patient can be effectively grasped, and the correct treatment method can be provided to the patient.

During the treatment process, for serious injuries that require emergency treatment, such as head trauma, chest trauma, and abdominal trauma, the patient must be sent to the operating room for surgical treatment in time [20]. Bleeding should be carefully controlled during surgery. Fractures are easy to repair. Use plaster to correct closed fractures of the upper and lower limbs, use external fixators to correct open fractures, use continuous tibial tuberosity to correct closed femoral fractures, and then receive ICU rescue. The main purpose of resuscitation is to treat the patient. Reheat to improve the blood coagulation mechanism of the patient, correct the parasites in the body, and avoid another blow to the body [21].

### 2.3. Image Enhancement Technology

On November 8, 1894, German physicists discovered X-rays and took the first photo in human history [22]. Take a line photo, then use the IP board to record the CR, collect and record the DR completely digitally, and then perform a computed tomography (CT) scan. The use of these technologies in medical diagnosis has undergone unwavering changes. The internal structure and pathological changes of the human body allowed by clinicians can be clearly and accurately observed without surgery [23]. This greatly reduces the suffering of patients and improves the efficiency of clinicians in diagnosing diseases. However, most medical imaging equipment can only acquire grayscale images for human body scanning. Because the human eyes have poor ability to recognize grayscale, a lot of information is lost, and doctors need to rely on black and white images and images at the time of diagnosis. Diagnose the imaging performance of the patient under the conditions of self-learning and anatomical understanding.

At present, the application of ordinary X-ray diagnosis can only be applied in mammography. There are no diagnostic reports on the chest, abdomen, or skeletal system. Due to the complex structure of breast tissue, it is very soft. In addition, mammography images are often copied, and mammography images, especially dense images of breasts, have no layers, resulting in a high rate of misdiagnosis and missed diagnosis. Previous reports [24] showed that the detection rate of typical mammography targets was less than 80%. For some asymptomatic breast cancers, the detection rate is even lower than 18%, and the misdiagnosis rate is high. Almost half of patients with suspected breast cancer will develop cancer during mammograms and will be misdiagnosed if they require further examination. In this report, through image enhancement technology, the detection rate of breast lesions has been significantly improved, more than half of the missed diagnosis patients can be diagnosed, and the misdiagnosis caused by uterine fibroids can almost be avoided [25]. It has been confirmed that image enhancement technology has important value in mammography diagnostic imaging.

The image enhancement technology based on the deep trust network model is also used for image processing, such as endoscopy, infrared imaging, and HIFU, and for determining the degree of tissue damage in orthopedic trauma. In the research of these applications, compared with traditional grayscale images, images processed by image enhancement technology can significantly improve the diagnosis of lesions.

The stability of the internal fixation must be ensured so that patients can exercise relative joint function as soon as possible after the fracture and reduce the associated postoperative complications. In addition to fracture classification, the choice of fracture treatment options should also take into account age. The presence or absence of fracture injury and the combination with other related comorbidities and the existence of fracture injury and other complications should also be taken into account. For younger patients, conservative treatment and surgical treatment will achieve better results. The former mainly includes incision skin necrosis. The latter seriously affects the lives of patients, including fracture deformities and traumatic arthritis. Therefore, in the surgical treatment of fractures, not only preoperative preparations must be made but also the correct surgical method and reduction of surgical trauma must be selected on the premise of restoring anatomical contraction, so as to improve the curative effect and reduce the suffering of patients. After treatment, related prognostic treatment should also be carried out to prevent various complications. The image enhancement technology based on the deep trust network model can also help patients with prognostic treatment and effectively reduce the difficulty of postoperative care.

## 3. Clinical Treatment Experiment of Trauma and Orthopedics

### 3.1. Research Objects

Collect fracture patients treated at the Department of Traumatology and Orthopedics of the First Hospital of the City from January 2019 to December 2020. Collect the fracture patients who were treated with traditional treatment methods from January 2019 to December 2020. According to the different treatment methods, the patients using the image enhancement technology of the deep trust network model are divided into the observation group (DCO group) and the patients using the traditional treatment method are divided into the control group (EDT group).

(1) Patient inclusion criteria:
  1. Injury severity score (InjurySeverityScore, ISS) ≥ 16 points
  2. The age is more than 15 years old
  3. Through imaging examinations of the patient's pelvis, spine, and limbs, the existence of fractures was confirmed
(2) Exclusion criteria:
  1. Fractures and dislocations caused by pathological fractures
  2. Those who are unable to judge or have incomplete information that affect the accuracy of the results
  3. Those who have mental illness or are pregnant

### 3.2. Baseline Data

1. Data content: collect the general information of the patient, such as age, gender, trauma severity score (ISS score), and cause of injury, and collect the total operation time, ICU resuscitation time, intraoperative blood loss, hospital stay during treatment of the patient, and the patient's death and complications.
2. Collection method: query the electronic medical record system of the city's first hospital, find qualified patient information based on the patient's clinical diagnosis and the above screening criteria, borrow patient medical records in the medical record room, view patient-related information, and collect patient-related information.

### 3.3. Observation Indicators

Compare the general conditions of the two groups (gender, age, ISS score, and cause of injury) to determine if there is comparability, compare the ICU recovery time of the two groups (d), postoperative blood transfusion (mL), total hospital stay (d), total operating time (min), postoperative complications (ARDS, MOF, postoperative infection, and DIC), and death.

### 3.4. Statistics

All data analysis in this article uses SPSS19.0. Statistical test uses two-sided test, significance is defined as 0.05, and *P* < 0.05 is considered significant. The statistical results are displayed as mean ± standard deviation (*x* ± SD). When the test data obeys the normal distribution, the double *T*-test is used for comparison within the group, and the independent sample *T*-test is used for comparison between the groups. If the regular distribution is not sufficient, two independent samples and two related samples will be used for inspection.

## 4. Experimental Analysis of Clinical Treatment of Trauma and Orthopedics

### 4.1. Comparison of Patient Age, Gender, and ISS Score

As shown in Table 1, comparing general conditions between the two groups, the patient's age and ISS score data conform to the normal distribution. Using the two independent sample *t*-test method, there is no significant statistical difference between the two groups (*P* > 0.05). There was no significant statistical difference between the two groups by the method of chi-square test (*P* > 0.05).

Comparing the causes of injury between the two groups using the *R* × *C* square table test, as 37.5% of the expected value is less than 5 and the minimum expected value is 2.84, the exact Fisher probability method is required, and it is concluded that there are no significant statistics on the cause of injury in both groups. The difference (*P* > 0.05) is shown in Table 2. The test results in Tables 1 and 2 show that the two sets of data are comparable.

Through the comparison of the treatment indicators of the two groups of patients, in the ICU recovery time, the average recovery time of the DCO group was 11 days, and the average of the EDT group was 17 days. Because the data of the two groups conformed to the normal distribution, the two independent sample *t*-tests showed that the data of the two groups are obvious. The statistical difference (*P* < 0.05) indicates that the image enhancement technology using the deep trust network model can quickly restore the patient's physiological function and reduce the length of ICU stay. In the comparison of intraoperative blood transfusion between the two groups, the average blood transfusion of the DCO group was 380 mL, and the average blood transfusion of the EDT group was nearly 600 mL. The blood transfusion of the injury control group was significantly lower than that of the early definitive surgery group, and through statistical analysis, the data of the two groups also had obvious statistics. The academic difference (*P* < 0.05) indicates that the image enhancement technology of the deep trust network model can reduce the patient's bleeding in the treatment of patients with fractures. This method is more conducive to the control of patients' bleeding. In the comparison of the total hospital stay and the operation time of the patients, there is no significant statistical difference between the two groups. The total operation time of the DCO group is slightly longer than that of the EDT group, which may be related to the staged treatment of the patients, as shown in Table 3:

Analyzing the data of the two groups with the continuous-adjusted chi-square test showed that the two groups had significant statistical differences (*P* < 0.05), indicating that the use of injury control orthopedics concepts can reduce the severity of postoperative complications in patients, but there was no significant difference in complications between the two groups. There is no significant statistical difference, which may be related to the small sample size, as shown in Table 4:

### 4.2. Traumatology and Orthopedics Treatment Methods

For orthopedic trauma, the current treatment methods include regular posture changes, special mattress decompression, adequate nutrient intake, antibiotics, and the image enhancement technology used in this article. We make statistics on the current treatment population, as shown in Figure 3.

From Figure 3, we can see that, at this stage, because the patient does not understand the condition of orthopedists, the choice of image enhancement technology is not the first choice because this method requires more steps and costs. The picture shows that the main injuries are car accidents and injuries during the fall. Because the limbs, pelvis, and spine are the main stress points in the case of body impact and compression, it is very easy to cause serious fractures, or even open fractures. In addition to fractures, patients often have injuries to other parts, mainly chest, abdomen, and brain injuries. The patient's hemodynamics is extremely unstable when admitted to the hospital, and severe fractures cause the fracture to the surrounding organs, skin, and soft tissues. And, major blood vessels cause damage, prone to traumatic hemorrhagic shock.

We have studied the images of patients' orthopedic trauma, as shown in Figure 4:

It can be seen from Figure 4 that the traumatic reaction leads to the systemic inflammatory response syndrome (SIRS), which leads to increased susceptibility. In addition, the serious pollution of open wounds and the long-term use of various invasive catheters increase the incidence of body infections. It is easy to cause infection of drug-resistant bacteria, resulting in the risk of ineffective antibiotic treatment. Through image enhancement technology, we can clearly understand the condition of the patient's fracture site. In the process of treatment, the image enhancement technology based on the deep trust model can effectively image the patient's injured site and understand the situation, as shown in Figure 5.

From Figure 5, we can see that, in the fractured part of the patient, through the image enhancement technology, the changes after the treatment can be clearly seen, which is conducive to the patient's rehabilitation and prognostic rehabilitation.

### 4.3. Prognostic Treatment

We look at statistics about the relevant parameters of patients before and after receiving treatment and compare the changes of patients before and after receiving treatment in order to understand the treatment effect, as shown in Figure 6:

From Figure 6, we can see that, after treatment, the patient's physical skills have improved significantly. Among them, the patient's blood supply and oxygen supply have been significantly improved, and the flexibility of the joints has been significantly improved. After 3 months of treatment, there is a clear contrast between traditional treatment and augmented reality technology. The treatment effect of image enhancement technology based on the trust network model is significantly better than the traditional treatment effect, and the patient's fracture site has been significantly improved.

We categorize trauma orthopedic patients, collect statistics on their living habits and physical conditions, and then conduct targeted rehabilitation and prognosis so that the patients can recover. The details are shown in Table 5:

From the table, we can see that poor living habits are an important reason for the slow prognosis of patients. Most patients have the habit of smoking and alcohol abuse, which causes the patients' own high blood fat and high blood pressure to be more serious, which greatly hinders rehabilitation of patients. We compare the rehabilitation prognosis of patients with normal schedules and patients with bad habits, as shown in Figure 7:

From Figure 7, we can see that compared with patients with normal work and rest, the recovery speed and efficiency of patients with poor work and rest is much lower, which shows that good living habits are extremely important for the prognosis and recovery of patients. In the rehabilitation of patients, attention should be paid to the patients' living habits in order to better recover the patients.

## 5. Conclusion

At the same time, there is the possibility of a fracture or fracture function, especially in cases with multiple fractures and a large injury, which may require a second treatment, which may cause damage to the elbow joint and increase the frequency of restriction of elbow joint movement. Image enhancement technology based on the deep trust network model can clearly understand the patient's condition and effectively prevent the formation of myositis. It can better restore bone strength, maintain the structural stability of the elbow joint and then maintain normal joint tension, which is beneficial for repairing the joint around the elbow joint, better maintain the stability of the elbow joint, and reduce the elevation of the bones caused by the fracture. And then, they cause symptoms like wrist pain. The research in this article also has some drawbacks. Due to limited equipment and research time, only this city's first hospital is used for data statistics. The sample has some limitations and will inevitably deviate from the actual situation in practical applications. This article hopes that more researchers can focus on the application of image enhancement technology in the clinical treatment of orthopedic trauma so that more accurate orthopedic trauma detection can be performed in the future.

## Figures and Tables

**Figure 1:** Deep trust network operation.

**Figure 2:** Flow chart of the deep trust network.

**Figure 3:** Number of people treated with pressure ulcers by different methods.

**Figure 4:** Comparison of fracture sites before and after surgery. (a) X-ray of femur and pelvis before surgery. (b) X-ray of femur and pelvis after surgery.

**Figure 5:** Partial imaging of the patient's fracture.

**Figure 6:** Before and after patient treatment. (a) Change after treatment. (b) 7 days after treatment. (c) After 1 month of treatment. (d) After 3 months of treatment.

**Figure 7:** Comparison of patients' prognosis and rehabilitation. (a) Normal patient. (b) Rehabilitation of patient with bad habits.

**Table 1:** Comparison of patient conditions.

Group	Number of cases	Age	Gender (male/female)	ISS score
EDT	30	40.57 ± 8.19	19/8	21.56 ± 3.96
DCO	27	37.33 ± 9.89	17/13	23.85 ± 4.61
Test value	—	*t* = 1.131	*X* ^2^ = 0.308	*t* = −1.72
*P*	—	0.214	0.47	0.065

**Table 2:** Causes of injury caused by patients.

Group	Number of cases	Cause of injury			
		Come down	Car accident	Extrusion	Heavy objects
EDT	30	10	10	4	3
DCO	27	9	12	6	3
Test value	—	—	0.605	—	—
*P*	—	—	0.84	—	—

**Table 3:** Patient treatment indicators.

Group	ICU recovery time	Intraoperative blood transfusion	Total operation time (min)	Hospitalization time (days)
DCO $\left(\bar{n}=27\right)$	11.03 ± 2.78	379.33 ± 109.41	257.04 ± 61.06	26.20 ± 3.83
EDT $\left(\bar{n}=30\right)$	16.27 ± 4.87	578.78 ± 185.6	245.67 ± 45.04	30.82 ± 3.42
Test value	5.418	−4.773	0.725	−4.825
*P*	<0.001	<0.001	0.456	0.47

**Table 4:** Complications of patients.

Group	Number of cases	Complications (cases)			
		Postoperative infection	ARDS	MOF	DIC
DCO $\left(\bar{n}=27\right)$	30	5	4	2	3
EDT $\left(\bar{n}=30\right)$	27	2	1	1	0
Test value	—	1.328			
*P*	—	1.0			

**Table 5:** Living habits of patients.

Risk factors	Cardiogenic infarction	Noncardiac infarction	Sum	*P* value
Age ≥ 75	35	21	56	0.038
Male	60	18	78	0.052
Smoking	34	9	43	0.032
Drinking	22	7	29	0.014
Hypertension	82	37	119	0.013
Diabetes	32	12	44	0.023
Hyperlipidemia	34	13	47	0.027
Hyperhomocysteinemia	46	24	70	0.095

## Data Availability

We do not have permission to share data from the data provider.
